The article "Fish Consumption Measured during Pregnancy and Risk of Cardiovascular Diseases Later in Life: An Observational Prospective Study" was published in 2011. Journal: PLoS One.

# Fish Consumption Measured during Pregnancy and Risk of Cardiovascular Diseases Later in Life: An Observational Prospective Study

**DOI:** 10.1371/journal.pone.0027330

**Published:** 2011-11-08

**Authors:** Marin Strøm, Erik L. Mortensen, Tine B. Henriksen, Sjurdur F. Olsen

**Affiliations:** 1 Maternal Nutrition Group, Department of Epidemiology Research, Statens Serum Institut, Copenhagen, Denmark; 2 Department of Environmental Health, Institute of Public Health and Center for Healthy Aging, University of Copenhagen, Copenhagen, Denmark; 3 Perinatal Epidemiology Research Unit, Department of Paediatrics, Aarhus University Hospital, Aarhus, Denmark; UCL Institute of Child Health, University College London, United Kingdom

## Abstract

Previous studies have indicated a protective effect of long chain *n*-3 PUFAs against cardiovascular disease; however, the overall evidence remains uncertain, and there is a general lack of knowledge in the field of cardiovascular epidemiology in women. Therefore, the objective of this study was to explore the association between fish intake and cardiovascular disease among 7429 women from a prospective pregnancy cohort in Aarhus, Denmark, who were followed for 12–17 years. Exposure information derived from a questionnaire sent to the women in gestation week 16, and daily fish consumption was quantified based on assumptions of standard portion sizes and food tables. Information on admissions to hospital was obtained from the Danish National Patient Registry and diagnoses of hypertensive, cerebrovascular and ischaemic heart disease were used to define the outcome: cardiovascular disease. During the follow-up period 263 events of cardiovascular disease were identified. Overall, there was no association between cardiovascular disease and fish intake, confidence intervals for effect estimates in the different fish intake groups were wide, overlapped and for all but one they encompassed unity. Restricting the analysis to women who had reported the same fish intake in a questionnaire in gestation week 30 did not alter these findings. In conclusion, our data from a prospective cohort of relatively young and initially healthy women from Aarhus linked with information from registries could not substantiate a protective effect of fish intake against cardiovascular disease.

## Introduction

Cardiovascular diseases are a serious public health concern worldwide. In Denmark more than 33000 persons are afflicted of ischaemic heart disease each year [1], and it has been estimated by the World Health Organisation that one third of all deaths are attributable to cardiovascular diseases [2].

Based on observations in the Greenland Inuit, where the incidence of coronary heart disease, and in particular acute myocardial infarction, was very low [3] a beneficial cardiovascular effect of the essential long chain *n*-3 PUFAs (LC*n*3FAs) has been hypothesized. Since then evidence from observational prospective studies [4]–[8] and randomized controlled trials [9]–[11] has supported this hypothesis of a protective effect of fish consumption and intake of, LC*n*3Fas that are obtained through fish consumption, against cardiovascular diseases. Also, a review assessing whether a valid association exists between dietary exposures and coronary heart disease in relation to the Bradford Hill guidelines reported moderate evidence for an effect of intake of fish and LC*n*3FAs [12]. However, a much debated Cochrane review from 2004 concluded that it is unclear whether dietary or supplemental LC*n*3FAs alter the risk of cardiovascular events on high risk or in the general population, but that there was no evidence to advise people to stop taking rich sources of LC*n*3FAs [13]. Likewise, a recent review of the cardiovascular effects of LC*n*3FAs concluded that while there is evidence of several beneficial cardiovascular effects of LC*n*3FAs there are still many uncertainties in the field, for example regarding risk of arrhytmic events [14], so the evidence in the field is still contradictory.

The article "Fish Consumption Measured during Pregnancy and Risk of Cardiovascular Diseases Later in Life: An Observational Prospective Study" was published in 2011. Journal: PLoS One.

Recently it has been emphasized by experts that women are underrepresented in cardiovascular research [15] and an overview of the literature reveals that there are few studies on effects of LC*n*3FAs in women. The large birth cohorts that have emerged in several countries in the last decade provide an opportunity for such observational studies. One of the main purposes of these cohorts was to investigate the significance of fetal or early exposures for development and health of the offspring. Nevertheless, the information collected on a wide range of maternal exposures and characteristics, including diet, facilitates studies on aetiological associations in the maternal population as well.

It can be argued that dietary intake during pregnancy might not reflect the habitual diet of an individual; however, during the recruitment period for this study (1992–1996) dietary recommendations regarding fish were the same as for the general populations. Furthermore, dietary patterns have previously been shown to be relatively persistent from preconception, through pregnancy and postpartum [16].

On this background the aim of the present study was to examine the relationship between fish consumption and the risk of cardiovascular disease approximately 12 years later in a Danish pregnancy cohort of relatively young and initially healthy women.

The article "Fish Consumption Measured during Pregnancy and Risk of Cardiovascular Diseases Later in Life: An Observational Prospective Study" was published in 2011. Journal: PLoS One.

In such a cohort a low number of cardiovascular events is expected, and therefore a mixed outcome is used, including cardiovascular diseases and the cardiovascular risk factor hypertension.

## Methods

### Ethics statement

The protocol for the study cohort was approved by the Central Denmark Region Committees on Biomedical Research Ethics. An informed consent form was used to obtain written consent from all participants.

Since 1990, and nearly consecutively until today, all Danish-speaking pregnant women attending routine antenatal care at the Department of Obstetrics and Gynaecology, Aarhus University Hospital, Denmark, have been invited to participate in the Aarhus Birth Cohort (ABC). The department serves all pregnant women in the area (high as well as low risk), and nearly all women in the area comply with the antenatal care programme [17]. The study base has been described in detail elsewhere [18], [19]. In short, women completed self-administered questionnaires in gestation weeks 16 and 30 regarding a range of medical, obstetric, demographic and behavioural factors. From September 1992 to October 1996 information on fish intake was part of the data collection and women who were enrolled during this period were included in the study population (N = 8729).

### Exposure

In Denmark fish is eaten mainly as part of a hot meal, open sandwich, or cold in a green or a pasta salad [20]. A previous study based on pregnant women from Aarhus has shown frequencies by which such meals are consumed to be strong and independent predictors of variation in erythrocyte *n*-3 fatty acids, without considering whether the meals contained fat or lean fish [20]. Four questions regarding fish consumption were therefore posed: How often did you eat (1) fish in a hot meal, (2) bread with fish, (3) green salad or pasta salad with fish, and (4) fish oil as a supplement. The women were asked to understand the term ‘fish’ as also comprising roe, prawn, crab and mussel. Each question had six predefined response categories: never, less than once per month, 1–3 times per month, 1–2 times per week, 3–6 times per week, every day.

In the week 16 questionnaire, women in the ABC were instructed to base their response on the period from when they knew they were pregnant until completing the questionnaire. In the week 30 questionnaire the women were asked to base their response on the period from around gestation week 16 until completing the week 30 questionnaire.

In the quantification of daily fish consumption we let the six different frequency categories correspond to: 0, 0.5, 2, 6, 18 and 28 servings per 28 days, respectively. Furthermore, we assumed that each serving of fish as a hot meal provided 144 g of fish, a fish sandwich provided 29 g of fish and a fish salad provided 50 g of fish. These values were mainly derived from work done by the Danish Veterinary and Food Administration on portion sizes, distributions of fish species in meals, and food tables for the Danish population [19], [21], [22]. We defined six exposure groups based on information from the week 16 questionnaire, with the lowest group comprising women who reported never eating fish, and dividing the remaining study participants into quintiles of daily fish intake. These exposure groups were decided upon a priori to enable us to investigate any possible effects in a null intake group, and still have a relatively large comparison group (the highest quintile).

The article "Fish Consumption Measured during Pregnancy and Risk of Cardiovascular Diseases Later in Life: An Observational Prospective Study" was published in 2011. Journal: PLoS One.

As a secondary exposure variable we combined the information from the 16 and 30 week questionnaires to obtain a measure of consistently reported fish consumption across the pregnancy period. We disregarded information on fish eaten with salad, since this contributed very little to the total fish intake. This measure was based on the subgroup of women who reported eating fish with the same frequency on both occasions. Furthermore, women consuming fish as a hot meal and as an open sandwich at different frequencies were excluded in order to obtain maximum contrast between the exposure groups. This did, along with the criteria of identical reporting in the two questionnaires, result in a marked restriction of the study sample (N = 650). To ensure a monotonously increasing exposure intensity across the exposure groups, women in this subsample were divided into the following categories, where both the defining variables increased progressively: fish consumption (hot meal and open sandwiches) on both measurement occasions (1) zero times, (2) more often, but less than once per month, (3) 1–3 times per month, and (4) once or more often per week.

### Outcome

We obtained information on all admissions to hospital regarding the study participants from the Danish National Patient Registry (NPR). The NPR contains information on all hospitalizations in Denmark since 1977 [23]. We assessed diagnosis of cerebrovascular diseases (International Classification of Diagnosis system 10 (ICD-10) codes I60-69, ICD-8 codes 430–438), ischaemic heart diseases (ICD-10 codes I20-25, ICD-8 codes 410–414), and hypertensive diseases (ICD-10 codes I10-15, ICD-8 codes 400–404). We defined an event of cardiovascular disease as a woman admitted to hospital with one of the diagnoses listed above, after terminating the pregnancy with which she entered the study population, and before the end of follow up, which was 1 December 2009.

The article "Fish Consumption Measured during Pregnancy and Risk of Cardiovascular Diseases Later in Life: An Observational Prospective Study" was published in 2011. Journal: PLoS One.

In supplementary analyses we investigated the associations between fish consumption and each of the endpoints: cerebrovascular, hypertensive and ischaemic heart disease, separately. Furthermore, we discerned between inpatient, outpatient and emergency room contacts and we used information on all diagnoses of cardiovascular disease prior to pregnancy.

### Covariates

From the questionnaires we gathered information on covariates used in the multivariable analyses. Based on the findings of previous studies in the field, we identified a priori and investigated the following variables as covariates: smoking prior to pregnancy (no, <10 cigarettes/day, >10 cigarettes/day), alcohol consumption during pregnancy (<1, 1–2, 3+ drinks per week), parity (0, 1+) prepregnant BMI treated as a continuous variable using restricted, cubic splines [24], cohabitant status (single, cohabitant), secondary education (no post secondary education, student while pregnant, <3, 3–4, >5 y post secondary education), school (<8, 8–9, >9 y school), gestational diabetes (no, yes according to NPR) and preeclampsia (no, yes according to NPR).

### Statistical analyses

A total of 8729 women were enrolled in the ABC between 1992–1996. We excluded women who reported taking fish oil as a supplement, yielding a study population of 8095 women. This was done to avoid the analytical difficulties of distinguishing between effects of food and supplement derived nutrients as we were not able to quantify intake of LC*n*3FAs from supplements. Further, a complete case analysis strategy was applied, and thus data from 7429 women was included in our final study sample. Women who entered our final study population were similar to those who were excluded with respect to age at enrolment, parity, smoking, BMI and cohabitant status.

Kaplan-Meier estimates of the survivor functions were investigated to characterize the effect of exposure. We used Cox regression models to investigate the risk of cardiovascular disease associated with different levels of fish consumption, while taking a number of covariates into account. Hazard ratios (HR) and 95% confidence intervals (CIs) were assessed, using age as the underlying time scale, and we applied delayed entry to account for the fact, that women entered the cohort at different ages. Participants were thus considered at risk from their age at the time when they filled in the week 16 questionnaire, until the age at cardiovascular disease diagnosis, death or the defined end of follow up, whichever came first. Investigation of the cumulative residuals did not reveal any violations to the assumption of proportional hazards. Trend tests for hazard ratios were performed by including the fish intake levels coded as 1, 2, 3, 4, 5, 6 and testing the significance of this variable.

The article "Fish Consumption Measured during Pregnancy and Risk of Cardiovascular Diseases Later in Life: An Observational Prospective Study" was published in 2011. Journal: PLoS One.

We adjusted for confounding by including the covariates smoking, alcohol consumption, parity, BMI, cohabitant status, education and school as explanatory variables simultaneously in the models. All analyses were carried out using SAS statistical software (version 9; SAS Institute, Cary, NC).

### Supplementary and sensitivity analyses

Supplementary analyses were performed to test the robustness of the findings. Using information on fish consumption from the week 30 questionnaire, we conducted analyses corresponding to the primary analyses. We also restricted the study population by excluding women who suffered from preeclampsia or gestational diabetes during the index pregnancy, as these might act as intermediate variables. Compared to diagnoses based on inpatient contacts, those based on emergency room and/or outpatient contacts may be less valid. In a sensitivity analysis we therefore excluded all events that were based on emergency room and/or outpatient contacts. Furthermore, individual analyses were conducted for each of the three endpoints (hypertensive, ischaemic and cerebrovascular disease).

## Results

Characteristics of the women in the study sample are given in table 1. During the follow up period from 1992/1997 – 2009 (median follow up time 15 years), 263 events of cardiovascular disease were identified in the study sample. Of these 154 were events of hypertension, 58 were events of cerebrovascular and 51 events of ischaemic heart disease.

**Table 1:** Participants in the Aarhus Birth Cohort distributed by maternal characteristics, fish intake in gestation week 16 and cardiovascular disease (CVD) (N = 7429).

	Overall		Fish intake g/day^a^							CVD^a^		
	N	All^a^	0	1^st^	2^nd^	3^rd^	4^th^	5^th^	*P* b	CVD	No CVD	*P* b
Maternal age (%)^c^									<0.0001			0.009
<20 y	68	1	7	2	1	0.2	0.5	0.4		0.4	0.9	
20–29 y	982	13	31	20	15	11	9	8		10	13	
30–39 y	3110	42	34	45	44	40	43	39		35	42	
40+y	3269	44	28	33	40	49	48	52		54	44	
Nulliparous (%)^c^	4240	57	64	63	60	55	53	53	<0.0001	47	57	0.001
Single/unmarried (%)^c^	322	4	8	5	5	4	3	5	0.0007	5	4	0.62
Nonsmokers (%)^c^	4855	65	50	60	65	69	67	69	<0.0001	66	63	0.04
Alcohol during pregnancy (%)^c^									<0.0001			0.2
<1 drink/week	5290	71	86	76	74	69	68	67		71	71	
1–2 drinks/week	1596	21	13	19	20	23	24	24		19	21	
>3 drinks/week	543	7	0.9	6	7	8	8	9		9	7	
Pre-pregnant body mass index (%)^c^									<0.0001			0.002
<18.5	465	6	8	6	8	5	6	6		8	6	
18.5–25	5795	78	69	74	75	81	78	82		69	78	
>25	1169	16	24	20	17	14	16	12		23	15	
School (%)^c^									<0.0001			0.001
<8 y	752	10	28	15	12	6	7	7		11	10	
8–9 y	2193	30	37	40	32	27	25	22		39	29	
>10 y	4484	60	35	45	57	67	68	71		50	61	
Secondary education (%)^c^									<0.0001			0.006
None	978	13	34	17	15	10	10	11		15	13	
3 y	2236	30	34	39	36	27	27	20		35	30	
>3–4 y	2544	34	17	28	31	38	36	40		37	34	
Student	944	13	10	10	10	13	14	17		7	13	
>4 y	727	10	5	6	8	12	12	12		6	10	
Preeclampsia (%)^c^	126	2	3	2	2	2	2	1	0.01	9	1	<0.0001
Gestational diabetes (%)^c^	8	0.1	0.4	0	0.1	0.1	0.1	0.1	0.52	0	0.1	0.57

a % (columns) of women distributed by covariate/covariate within level of exposure or outcome.

b Two-sided *p*-value from χ2-test for measure of association.

c % (columns) of women within fish intake group.

The article "Fish Consumption Measured during Pregnancy and Risk of Cardiovascular Diseases Later in Life: An Observational Prospective Study" was published in 2011. Journal: PLoS One.

Women with a low fish intake were more likely to be young (<30 y), nulliparous, smokers, overweight, have a low alcohol intake, be less educated and more likely to suffer from preeclampsia as compared to women with a high fish intake. Among women who suffered from cardiovascular disease there were more women who were older at recruitment, parous, smoking, overweight, less educated and there were more preeclampsia cases than among women who did not suffer from cardiovascular disease during the study period (table 1).

Table 2 shows crude and adjusted HRs for cardiovascular disease, with women in the highest fish intake group as the reference group. For women in the 2^nd^ quintile of fish intake (median intake 8 g/day) there was an increased risk of cardiovascular disease adjusted HR 1.54 (95% CI 1.03, 2.28). Regarding women in lower and higher fish intake groups risk estimates were closer to one and CIs encompassed unity. Overall, there was no association between cardiovascular disease and fish intake, either when the latter was treated as a categorical (*p* = 0.29) or as a continuous variable (*p* = 0.97).

**Table 2:** Hazard ratios (HRs) for risk of cardiovascular disease according to fish intake among 7429 women in the Aarhus Birth Cohort.

			Cardiovascular disease				
Intake of fish			No. of cases	Crude		Adjusted^a^	
(mean g/day)	N	%		HR	95%CI	HR	95%CI
No fish intake (0)	235	3	5	0.99	(0.39–2.51)	0.77	(0.30–1.96)
Lowest quintile (3)	1470	20	49	1.38	(0.91–2.08)	1.12	(0.74–1.71)
Second quintile (8)	1404	19	62	1.73	(1.17–2.56)	1.53	(1.03–2.27)
Third quintile (13)	1609	22	57	1.23	(0.83–1.83)	1.19	(0.80–1.77)
Fourth quintile (18)	1280	17	48	1.32	(0.87–1.99)	1.27	(0.84–1.92)
Highest quintile (39)	1431	19	42	Ref	-	Ref	-
					p = 0.13^b^		p = 0.28^b^
					p = 0.09^c^		p = 0.61^c^

HR, hazard ratio; CI, confidence interval.

a Adjusted for smoking, alcohol intake, parity, cohabitant status, school, education and prepregnant body mass index.

b Over-all χ2-test of effects.

c Test for trend.

The analysis in table 3 is based on the subgroup of women who consistently reported the same frequency of fish intake in the week 16 and 30 questionnaires, restricting the study sample substantially. No association between this exposure measure and risk of cardiovascular disease was seen, adjusted HRs ranging from 0.98 (95% CI: 0.22, 4.34) to 1.92 (95% CI: 0.53, 7.04).

The article "Fish Consumption Measured during Pregnancy and Risk of Cardiovascular Diseases Later in Life: An Observational Prospective Study" was published in 2011. Journal: PLoS One.

**Table 3:** Hazard ratios (HRs) for risk of cardiovascular disease according to fish intake among 650 women in the Aarhus Birth Cohort, who consistently reported the same fish intake in 1st and 2nd trimester.

			Cardiovascular disease				
			No. of Cases	Crude		Adjusted^a^	
Intake of fish	N	%		HR	95%CI	HR	95%CI
Zero intake	139	21	4	1.35	(0.33–5.49)	0.95	(0.20–4.41)
<Each month	127	19	8	2.15	(0.65–7.15)	2.03	(0.55–7.53)
Each month	271	42	12	1.34	(0.43–4.16)	1.26	(0.39–4.03)
Each week	113	17	4	Ref	-	Ref	-
					p = 0.60^b^		p = 0.57^b^
					p = 0.44^c^		p = 0.88 c

HR, hazard ratio; CI, confidence interval.

a Adjusted for smoking, alcohol intake, parity, cohabitant status, school, education and prepregnant body mass index.

b Over-all χ2-test of effects.

c Test for trend.

Shifting the exposure to fish intake from the week 30 questionnaire did not change these findings, and neither did: 1) applying a different categorisation of fish intake (no fish intake/lowest quintile/three middle quintiles (ref.)/highest quintile); 2) an exclusion of women who had preeclampsia or gestational diabetes during the index pregnancy; 3) exclusion of outpatient and/or emergency room contact based events; or 4) using the three endpoints as individual outcomes (data for supplementary analyses not shown).

## Discussion

In our study population of relatively young and initially healthy Danish women, there was no clear evidence of an association between fish intake measured during pregnancy and subsequent risk of cardiovascular disease.

The biological properties of LC*n*3FAs and the pathophysiology of cardiovascular disease make the idea of a protective effect of seafood consumption against cardiovascular disease probable. Physiological effects of intake of LCn3FAs include altered cell membrane fluidity and receptor responses following incorporation of LCn3FAs into cell membrane phospholipids [25], [26], as well as direct binding of LCn3FAs to cytosolic receptors that regulate gene transcription [27] and complex interactions with ion channels [28]. These mechanisms have varying dose-responses and time-responses of effect [29]. Apparent discrepancies in the results of previous studies might thus reflect the different responses of effect depending upon the chosen outcome measure, as well as differences in levels of habitual intake across study populations. Furthermore, although most cardiovascular risk factors are shared by men and women, there might be gender differences with regard to their impact [30], and inflammation, HDL and triglyceride levels might have a more negative influence on cardiovascular risk in women than in men [30]. Since these risk factors are supposedly affected by LCn3FA intake, this underlines a need for studies on the importance of LCn3FAs in women.

The article "Fish Consumption Measured during Pregnancy and Risk of Cardiovascular Diseases Later in Life: An Observational Prospective Study" was published in 2011. Journal: PLoS One.

### Comparison with other studies

The setting of our study in a pregnancy cohort implied that participants were generally young and healthy at enrolment. These demographic characteristics and the composite outcome definition in our study complicate comparisons with other studies in the field.

Most of the randomized controlled trials that have been conducted in this field have been secondary prevention trials conducted in male study populations [9]–[11]. Several observational prospective studies have shown fish consumption and LC*n*3FAs in varying amounts to be inversely associated with fatal coronary heart disease [4]–[8]. In some observational studies no such association has been observed [31]–[33], or an association has been seen for some, but not for other cardiovascular outcomes [34]. These inconsistencies are also reflected in the different reviews that have been conducted in this area of research. In a review on health effects associated with consumption of fish and the contaminants that come along with it, the authors concluded that the health benefits of fish intake outweigh risks emanating from methylmercury, dioxins and PCBs [35]. Likewise, some reviews have concluded that there is solid evidence of a protective effect of LC*n*3FAs against cardiovascular mortality [29], [36], [37], while others seem to unveil a more complex picture [13], [14].

Only few studies have been carried out in female study populations. Another recent Danish follow-up study including middle-aged men and women showed an inverse association between intake of fatty fish and risk of acute coronary syndrome in men, but no association in women [38]. This finding is in accordance with our study, but stands in contrast to the results from a large observational prospective cohort of women, the Nurses' Health Study, where intake of fish and LCn3FAs was found to be inversely associated with risk of coronary heart disease [39] and thrombotic infarction [40].

Most previous studies have been carried out in populations that were older compared to the ABC, and many have modelled cardiovascular mortality rather than risk of incident events. This might be the reason why our findings seem to stand in contrast to many other studies in the field.

The article "Fish Consumption Measured during Pregnancy and Risk of Cardiovascular Diseases Later in Life: An Observational Prospective Study" was published in 2011. Journal: PLoS One.

### Strengths and weaknesses of the study

The major strengths of our study are its prospective design, the close-to-complete follow up from high quality registry data and the relatively detailed information on fish intake during pregnancy. The fish intake questions have earlier been validated against biomarkers in the study population (pregnant women in Aarhus). A comparison of intake of LC*n*3FAs, estimated by a combined dietary self-administered questionnaire and interview, with fatty acids measured in erythrocyte phospholipids showed that with respect to the power to explain FA-ratio variability, the questions on fish consumption used in our study were comparable with intake of LC*n*3FAs assessed by an elaborate semiquantitative dietary method involving an interview [20]. Furthermore, we had data on fish consumption for two separate periods of pregnancy enabling us to focus on a restricted study sample who consistently reported the same fish intake during 2nd and 3rd trimester, and we were able to adjust for some important potential confounding factors. Information on fish intake during pregnancy may be taken as an estimate of the habitual intake of the study participants, as dietary patterns have previously been shown to be relatively persistent from preconception, through pregnancy and postpartum [16], [41]. The most frequently consumed fish species in Denmark are cod, plaice, salmon herring, and mackerel, whereas species with high mercury content, such as shark and king mackerel, are not commonly consumed in Denmark [42]. Furthermore, during recruitment and initial data collection for the ABC dietary recommendations in Denmark did not include warnings regarding intake of fatty fish due to the potential harm of dioxins or methyl-mercury. Therefore it is less likely that women in the ABC have changed their fish intake during pregnancy either due to worries regarding harmful exposures, or due to considerations of beneficial effects of LC*n*3FAs to the developing fetus.

However, the information on nutrition did not comprise data on type of fish consumed, total energy intake or other dietary factors, such as meat, fruit and vegetables, trans fatty acids and n-6 polyunsaturated fatty acids, which have also been associated with cardiovascular disease. Since we are not able to disentangle dietary intake of LC*n*3FAs from that of overall fish consumption this might blur a potential underlying association between LCn3FAs and cardiovascular diseases. Furthermore, we are not able to adjust for some known dietary risk factors for cardiovascular diseases, such as trans-fatty acids; and – as in any observational study - we cannot exclude residual confounding or confounding by factors not adjusted for.

The article "Fish Consumption Measured during Pregnancy and Risk of Cardiovascular Diseases Later in Life: An Observational Prospective Study" was published in 2011. Journal: PLoS One.

In table 2 an increased risk of cardiovascular disease for women with median fish intake of 8 g/day is observed. Either this finding reflects an underlying increased risk of cardiovascular disease for women who consume moderate vs high amounts of fish; or the increased risk observed for the intermediate fish intake group is a chance finding, or reflecting residual confounding. An increased risk of cardiovascular disease related to moderate fish intake could result from consumption of the fish types that are high in environmental contaminants, and that positive effects of LC*n*3FAs would exceed the negative effects of contaminants only at the very highest fish intakes. However, this is largely speculative, and we find it more likely that the increased risk observed for the intermediate fish intake group is a chance finding, as indicated by the p-value for the overall χ^2^-test of effects.

Our results are in line with a previous Danish study which also included women in the study population, but both studies seem to suffer under a low number of cases. Therefore it is unclear wether our results are actually reflecting that there is no association between fish intake and risk of CVD in these relatively young Danish women, or whether the number of cases is simply too low to be used as the basis for any biologically relevant conclusions.

All pregnant women in Aarhus in the recruitment period were invited to participate in the ABC, but since it was not registered who did not participate the actual participation rate is not known, although it is estimated to be 76–95% for the different questionnaires [43]. It is generally assumed that persons who participate in large cohort studies are more health-conscious compared to non-participants; a selection that might result in biased effect estimates if the likelihood of being followed in the cohort depends on both the exposure and the outcome, or bias might be more subtly related to factors that influence exposure and outcome. Provided that the confounding which may have been introduced by the selection processes, is captured by the covariate models we used, selection may not be problem. Further, we believe that the same biological effects apply to the selected cohort as to the target population to which we want to generalize our results.

Preeclampsia, gestational diabetes and cardiovascular disease may share a common aetiology, or these pregnancy complications may be on the causal pathway to cardiovascular disease. Furthermore, women suffering from these conditions are often advised by health personnel to change their diet, and their report on fish intake during pregnancy might thus not be a valid estimate of their habitual intake. However, excluding women who had suffered from preeclampsia and gestational diabetes during the index pregnancy did not alter our findings.

The article "Fish Consumption Measured during Pregnancy and Risk of Cardiovascular Diseases Later in Life: An Observational Prospective Study" was published in 2011. Journal: PLoS One.

Due to the demographic characteristics of the population we expected rates of mortality and coronary heart disease to be low. The validity of acute myocardial infarction in the NPR has previously been examined and found to be good [44], but we expected a low number of diagnoses of this disease among women in the ABC. Given these circumstances we chose to investigate a relatively broad range of cardiovascular diagnoses including hypertension, which is actually a risk factor for atherosclerosis. Subsequently, supplementary analyses were conducted where hypertensive, cerebrovascular and ischaemic heart disease were treated as individual outcomes, but this did not alter our conclusions.

Emergency room and outpatient contacts have been included in the NPR since 1995, but the validity of these diagnoses has been found to be lower than for other hospital departments[45]. Therefore, in a supplementary analysis, we excluded all emergency room or outpatient contacts but our results remained unchanged.

In the planning of this study estimations were performed regarding the expected number of cases of cardiovascular disease in the cohort and the power to detect differences in cardiovascular disease risk between exposure groups. This was done based on age and sex specific incidences of cardiovascular disease from ‘Heart Statistics’ [1]. Given the exposure groups used in this study power was calculated to be an acceptable 75% for detecting a difference in risk estimate of 30% (corresponding to the difference observed in a study on intake of fish/LC*n*3FAs and the risk of coronary heart disease in women by Hu et al [39]). However, it is well known that people who are socioeconomically advantaged are more likely to participate in cohort studies such as the ABC. Therefore the number of identified events of cardiovascular disease in our study was even lower than expected, and a potential association between fish consumption and cardiovascular disease may thus have been attenuated. In a relatively young study population such as the ABC early markers of cardiovascular disease, including blood cholesterol, blood pressure or micro-albuminuria, might be a better outcome measure; unfortunately, this information was not available.

### Conclusion

In conclusion, our data from a prospective cohort of women who were followed up for 15 years through high-quality registries could not substantiate a protective effect of fish intake against cardiovascular disease. Since the incidence of cardiovascular disease is low in women below 50 years further studies should be carried out in larger study populations or with early markers of cardiovascular disease as an outcome measure.
